RETRACTED

# The correlation between microvessel pathological changes of the endplate and degeneration of the intervertebral disc in diabetic rats

**DOI:** 10.3892/etm.2012.868

**Published:** 2012-12-20

**Authors:** SEN CHEN, MEIMEI LIAO, JIANPING LI, HAO PENG, MIN XIONG

**Affiliations:** 1 Department of Orthopedics, Renmin Hospital of Wuhan University, Wuhan, Hubei 430060;; 2 Dongfeng General Hospital, Hubei University of Medicine, Shiyan, Hubei 442008, P.R. China

**Keywords:** diabetes mellitus, intervertebral disc, microvessel

## Abstract

In this study, the pathological microvessel changes to the endplate and the degeneration of the intervertebral disc of diabetic rats were examined in order to identify the possible mechanism by which diabetes mellitus (DM) induces degeneration of the intervertebral disc. A total of 30 Sprague-Dawley rats were randomly divided into two groups. DM was induced in one of the groups by streptozotocin (STZ) administration. The rats were sacrificed 4, 8 and 12 weeks later. Five rats from each group were sacrificed at each time interval and lumbar disc and endplate tissue were obtained from each rat. The histological changes, collagen expression, microvessel density (MVD) and apoptosis of the disc were investigated by different methods. The expression of collagen I in the diabetic DM group was higher compared to the control group at the three time points (P<0.01), in contrast to the expression of collagen II. The factor VIII-related antigen (FVIII RAg) was expressed in the control and DM groups, while its expression was relatively low in the DM group. The MVD of the DM group was smaller compared to that of the control group at the three time points (P<0.01). The apoptotic index (AI) in the diabetic group was significantly higher compared to that of the control group at the three time points (P<0.01). A negative correlation was observed between the MVD of the endplates and the notochordal cell AI in the two groups. Compared to the control group, the endplate MVD decreased and the cavity became smaller or disappeared in the diabetic rats. In conclusion, there was a negative correlation between MVD and degenerative changes of the intervertebral disc in diabetic rats.

## Introduction

Diabetes mellitus (DM) is a systemic endocrine and metabolic disease with chronic complications that damages almost every organ and system of the body (1–5). One of the characteristic complications of DM is microangiopathy, which constitutes the pathophysiological basis of a wide range of organ damage. In addition to causing diabetic retinopathy, nephropathy and cardiomyopathy, diabetic microangiopathy damages the inter-vertebral disc (6–11). Although the disc is avascular, it depends on diffusion from microvessels at the endplate of the disc to supply the nutrients essential for cell activity and viability and to remove metabolic wastes (12–14). Changes in blood supply cause a deficiency of nutrient supply (10,15–18). This study examined the pathological microvessel changes to the endplate and the degeneration of the intervertebral disc in diabetic rats in order to identify the possible mechanism by which DM induces degeneration of intervertebral discs.

RETRACTED

## Materials and methods

### Animals

A total of 30, three-month-old male adult Sprague-Dawley (SD) rats, obtained from the Experimental Animal Center of Wuhan University, Wuhan, China, and weighing 231–263 g, were used in this study. The rats were housed 5/cage under standard laboratory conditions (12/12-h light/dark cycle, at a temperature of 24–25°C and humidity of 50–55%) and allowed free access to food and water during the study. The rats were fed on a normal pellet diet. All the experimental protocols adhered to the Guidelines for the Care and Use of Laboratory Animals published by the U.S. National Institutes of Health (NIH Publication, revised 1996). The study was approved by the Ethics Committee for Animal Research of Wuhan University, (Wuhan, China).

### Grouping and treatment

The rats were randomly divided into the streptozotocin (STZ)-induced diabetes group (DM) and the control group (n=15 rats/group). The fasting blood glucose was measured by examining blood samples from the tail vein using a rapid blood glucose meter (One Touch II; Johnson & Johnson, New Brunswick, NJ, USA). DM was then induced by a single intraperitoneal (i.p.) injection of STZ solution (50 mg/kg). In the control group, the rats were administered the same volume of sodium citrate buffer. Fasting blood glucose levels were measured 3 days later. The blood glucose was examined ≥3 times following STZ injection and every two weeks thereafter. The standard glucose measurement for the diagnosis of DM was >13.8 mmol/l. The rats were sacrificed with a lethal dose of sodium pentobarbital (60 mg/kg i.p.) at intervals of 4, 8 and 12 weeks later. Five rats in each group were sacrificed at each time interval and lumbar disc tissue and endplate was obtained from each rat.

### Histopathology

The lumbar 5/6 disc was fixed in 4% para-formaldehyde-0.1 M phosphate buffer (pH 7.4), followed by decalcification with 10% ethylenediaminetetraacetic acid (EDTA)-0.1 M phosphate buffer (pH 7.4). Following decalcification, the tissues were dehydrated in graded ethanol, embedded in paraffin, cut into 6-*μ*m sections in the coronal plane and processed for routine hematoxylin and eosin staining for the evaluation of degeneration under a light microscope. The sections were assessed blindly by two independent authors.

RETRACTED

### Ultrastructure observation

At 12 weeks, two rats were randomly selected from each group for ultrastructure observation. The lumbar 2/3 disc was fixed with 3% glutaraldehyde solution and then sent to the Microscope Center of Wuhan University for ultrastructure observation.

### Immunohistochemistry

Immunohistochemical staining was conducted using the streptavidin-peroxidase complex method. Rabbit anti-mouse collagen I and II, and the factor VIII- related antigen (FVIII RAg) (dilution, 1:200) (Santa Cruz Biotechnology Inc., Santa Cruz, CA, USA) polyclonal antibody was used as the primary antibody. Color development was achieved with 3,3′-diaminobenzidine (DAB), which stained positive cells brown. Cells with brown particles in the plasma were evaluated as positive results. Five views of each slice were randomly selected for analysis. Images were captured on a Zeiss Axioskop 40 microscope equipped with a Canon Eos 10D digital camera (Canon, New York, NY, USA). The optical density of collagen I and II was analyzed by a high resolution graphic analysis system and the average optical density of the five views was recorded as the expression of collagen in the sample.

### Microvessel density (MVD)

Microvessels were immunohistochemically marked by FVIII RAg staining. Positive results were determined by Weidner’s method (19). After screening the areas with microvessel spots at low-power field (magnification, ×100), microvessels in the area were counted in a ×400 field. Five separate areas were assessed and the mean was calculated to determine the MVD of each section.

### Appotosis of notochordal cells

Apoptotic notochordal cells were detected using the TUNEL method, with an *in situ* cell death detection kit (Roche Diagnostics, Mannheim, Germany). The assay was performed according to the manufacturer’s instructions. Briefly, following routine deparaffinization and treatment with H_2_O_2_ (3%), sections were digested with proteinase K (20 *μ*g/ml, pH 7.4, 12 min) at 25°C and incubated with the reaction mixture (1:40, 60 min) at 37°C. Incorporated fluorescein was detected with horseradish peroxidase following a 30-min incubation at 37°C and subsequently dyed with DAB. Brown nuclei were assessed as positive apoptotic cells. The apoptotic index (AI) was evaluated for one section of 5 high-power fields.

### Statistical analysis

Data were presented as the mean ± standard error of the mean. Statistical analysis was performed using SPSS 13.0 software (SPSS, Inc., Chicago, IL, USA). One-way analysis of variance (ANOVA) with Tukey’s post hoc test was used to examine differences between groups. The correlation between the endplate MVD and the nucleus pulposus cell AI was examined by Pearson’s correlation analysis. P<0.01 was considered to indicate a statistically significant difference.

RETRACTED

## Results

### Body weight and serum glucose levels

No accidental deaths occurred during the experiment. The STZ-induced diabetic rats showed significantly smaller body weights compared to the control animals. The typical symptoms of DM in the rats were polydypsia, polyphagia, polyuria and emaciation. The data presented in this study are the blood glucose measurement obtained the third time after the STZ injection. Following STZ injection, the serum glucose levels in the DM group were significantly higher compared to those in the control group (P<0.01) (Table I).

### Histological investigation

The histological structure of the disc appeared to be normal at 4, 8 and 12 weeks in the control group (Fig. 1A, C and E). Numerous microvessels were evident in the endplate. The discs of the controls consisted of a large amount of extracellular matrix interspersed with a small number of cells comprising ∼1% of the total volume, where cell morphology varied. Those in the annulus fibrosus and cartilage endplate were more elongated and fibroblast-like compared to those of the nucleus pulposus, which were more rounded or oval and chondrocyte-like, sometimes with a capsule around them. Misalignment was not observed in the inner or intermediate layers of the annulus fibrosus. Cracks and tears were also not observed.

By contrast, in the DM group, the histological structure of the discs gradually exhibited more degeneration at 4, 8 and 12 weeks (Fig. 1B, D and F). Fewer microvessels were evident in the endplate compared to the control group. Decreases in notochordal cells and increases in fibroblasts were observed. Enlarged chondrocytes were observed in the inner and intermediate layers of the annulus fibrosus. The annulus fibrosus demonstrated disrupted alignment and formation. There was also a reduction in the nucleus pulposus matrix accompanied by fibrosis and hyalinization, suggesting depletion of the extra-cellular matrix.

### Electron microscopic findings

In the control group, organ-elles such as the golgi apparatus, mitochondria, lysosomes and the cell membrane were intact and orderly with abundant glycogenosome and sparse lipid droplets in the plasma (Fig. 2A and C). Collagenous fibers were scattered neatly and closely in the plasma, while the mesh between the fibers was relatively small. The ultrastructure of the notochordal cell was different between the control and DM groups (Fig. 2B and D). The membrane of the cell and organelles was disrupted, while the organelles swelled and vacuolized and the nucleus structure was destroyed. Collagenous fibers were scattered loosely and messily in the plasma, while the meshes between the fibers were relatively large.

RETRACTED

### Expression of collagen I and II

The optical density of collagen I and II was used to perform a semi-quantitative analysis (Figs. 3 and 4). It was found that the collagen composition changed greatly in the nucleus pulposus, such that the proportion of collagen I increased, while the proportion of collagen II decreased. The results showed that the expression of collagen I in the diabetic group was higher compared to the control at the three time points (P<0.01) (Table II). However, the expression of collagen II in the DM group was lower compared to the control group at the three time points (P<0.01) (Table III).

### MVD of the endplates

FVIII RAg was selected as a marker of vascular endothelial cells to reveal the microvessels of the endplates. FVIII Rag was expressed in the control and DM groups, although the expression in the DM group was relatively low. MVD decreased in the two groups over time. The MVD of the DM group was smaller compared to that of the control group at the three time points (P<0.01) (Table IV).

### AI of notochordal cells

AI was measured by TUNEL assay (Fig. 5). A brown nucleus was assessed to be a positive apoptotic cell. Cell apoptosis occurred in the two groups. There were more apoptotic cells/high-power field in the DM group compared to the control group. AI increased over time in the two groups. AI in the diabetic group was significantly higher compared to the control group at the three time points (P<0.01) (Table V).

### Correlation analysis between MVD and notochordal cell AI

A decrease in MVD occurred while AI of the disc increased over time in the two groups. A negative correlation was observed between the endplate MVD and the notochordal cell AI in the control group (Pearson’s correlation coefficient, r=−0.953, P<0.01) (Fig. 6A). The same was observed in the DM group, with a correlation coefficient of −0.936 (P<0.01) (Fig. 6B).

## Discussion

There are two major nutrient transportation pathways in the intervertebral disc. One is the endplate pathway by which nutrients pass through the bone marrow cavity-blood sinus-cartilage endplate route to support the nucleus pulposus. The other is the annulus pathway. Previous studies have suggested that the endplate route is the major pathway for nutrient transfer to the intervertebral disc (20,21). There is a significant decrease in cortex thickness over the central portion of endplates and shells, with a mean minimum thickness of 0.40 mm, a mean maximum thickness of 0.86 mm and an overall mean of 0.64±0.41 mm. Increased porosity is also observed along the central regions of the cortical shells (22). The porous structure accounts for ∼7–10% of the endplate area (23), providing direct contact between the vertebral blood sinus and the endplate. There is a continuous capillary bed that is most dense in the area adjacent to the nucleus pulposus. There are a number of microvessel plexuses in the center with less MVD at the boundary (24). The vascular branches issuing from the microvessel plexuses pass through the porous structure and form microvessel buds in the endplate (25). These vessels drain either into the subchondral post-capillary venous network or directly into the veins of the marrow spaces in the vertebral bodies (26). The decrease in nutrients constituent in the disc is considered a key factor in disc degeneration (27–29). Loss of nutrient supply may lead to cell death, loss of matrix production and increase in matrix degradation, eventually leading to disc degeneration (10).

RETRACTED

The changes of collagen, proteoglycan and water content are the pathological characteristics of intervertebral disc degeneration caused by the dysfunction and quantitative reduction of the disc cells (7,23,29). The collagen ingredient changes that occur during the degeneration process include the decrease of collagen II and the increase of collagen I. A positive correlation reportedly exists between the amount of collagen reduction and the degree of intervertebral disc degeneration (30,31). The reason for the decrease in cell density is cell apoptosis, which is thought to be the principal cause of the extracellular matrix degradation (32,33). However, a high inverse correlation between the density of openings in the osseous endplate (in particular the size of the capillary buds) and the morphologic degeneration grade of the disc, supports the hypothesis that occlusion of these openings may deprive the cells of nutrients, leading to insufficient maintenance of the extracellular matrix and disc degeneration (15,34,35).

In this study, the expression of collagen I increased along with the progression of DM. When compared to the control, the difference was significant (P<0.01). The expression of collagen II follows the opposite pattern, decreasing with the progression of DM. In this instance, the difference between the experimental and the control groups was also significant (P<0.01). In addition, this study has demonstrated that the disc cell AI in the DM group was significantly higher compared to the control group (P<0.01).

Microangiopathy is one of the characteristic complications of DM and the pathophysiological basis of multi-organ damage. In this study, the pathological changes of microvessels in the endplate increased over time in the DM group. The cavity of the microvessels became smaller and less dense. When compared to the control, the difference was significant. The AI of the DM group was also significantly higher compared to the control group, resulting in changes in the extracellular matrix that included the decrease of collagen II and the increase of collagen I. The difference was statistically significant compared to the control (P <0.01). The histological findings confirmed the observations that the disc degeneration of the DM rats was greater compared to that of the control. The statistical analysis demonstrated a negative correlation between the endplate MVD and the notochordal cell AI in the DM and control groups.

RETRACTED

It can be hypothesized that hyperglycemia, low oxidative stress and advanced glycosylation end products in DM rats would cause microvessel endothelial cell injury of the disc endplates, thereby leading to either occlusion or a decrease in the number of microvessels. In the immediate aftermath, the blood supply of the disc would decline sharply, causing damage to the disc in two major ways. First, the disc nutrition would be decreased or lost entirely. Second, cellular metabolic wastes and toxins would not be able to be excreted and would accumulate in the disc leading to ischemia, hypoxia, acidosis and eventually to cell necrosis and apoptosis. Cell products would also change. The contents of proteglycan, collagen II and water would decrease, while the contents of collagen I would increase. Calcification and disc fissures would occur and the mechanical properties of the disc would degrade.

Limitations in using a rat lumbar disc model include a smaller disc size and a different cell composition of the rat lumbar disc compared to a human disc. In addition, unlike the human disc, the rat disc is subjected to less mechanical load as it stands on four legs. Due to the limited applicability of the rat model, experiments are necessary to determine the pathological changes of the disc in human beings suffering from DM.

In conclusion, compared to the control, the endplate MVD decreased and the cavity became small or disappeared in the DM rat. DM accelerated the degeneration process of the disc. The results of this study have shown that a negative correlation exists between the mircrovessel density and the degenerative changes of the intervertebral disc within diabetic rats. The aforementioned limitations should be taken into consideration when extrapolating the results to humans.

## Figures and Tables

**Figure 1.** Photomicrographs showing histological analysis of the transected disc samples. Hematoxylin and eosin (H&E) staining: (A), (C) and (E) show the apparently normal histological structure of the disc at 4, 8 and 12 weeks in the control group. (B), (D) and (F) show the histological structure of the discs exhibiting a gradual degeneration process at the different time points. Arrows in (B) and (D) show a reduction in notochordal cells. The arrow in (F) shows the disruption of the annulus fibrosus. Original magnification, ×100.

RETRACTED

**Figure 2.** The ultrastructure of the disc by scanning electron microscopy (SEM). (A) and (C) show the ultrastructure of the apparently normal disc at 12 weeks in the control group. (B) and (D) show the poor the performance of the discs in the DM group at 12 weeks. The arrow in (B) shows swelled organelles and incomplete nucleus. The arrow in (D) shows that the fibers were in disarray. Original magnification, ×6,000.

**Figure 3.** Photomicrographs showing the expression of collagen I in the disc samples. Immunohistochemical staining was used to show collagen I in the disc: (A), (C) and (E) show that the expression of collagen I was not significantly changed. (B), (D) and (F) show that the expression of collagen I significantly increased over time. Original magnification, ×400.

**Figure 4.** Photomicrographs showing the expression of collagen II in the disc samples. Immunohistochemical staining was used to show collagen I in the disc: (A), (C) and (E) show that the expression of collagen II was not significantly changed. (B), (D) and (F) show that the expression of collagen II significantly decreased over time. Original magnification, ×400.

**Figure 5.** Photomicrographs showing cell apoptosis in the disc samples. TUNEL staining was used to investigate the cell apoptosis of the disc at 12 weeks. The arrow indicates an apoptotic cell. Original magnification, ×400.

**Figure 6.** Images showing the correlation between the microvessel density (MVD) of the endplates and the notochordal cell apoptotic index (AI). There was a negative correlation between the MVD of the endplates and the notochordal cell AI in the (A) control and (B) DM groups.

**Table I.** Blood glucose of the rats of each group.

Group	Before injection	After injection
Control	5.21±0.696	5.13±0.464
DM	5.31±0.519^a^	20.27±2.600^b^

a P>0.01 and

b P<0.01 compared to the corresponding value in the control group. DM, diabetes mellitus.

**Table II.** Optical density of collagen I in the disc of each group.

Group	4 weeks	8 weeks	12 weeks
Control	0.1547±0.00765	0.1710±0.01117	0.1799±0.01395
DM	0.2783±0.01258^a^	0.4535±0.07003^a^	0.6078±0.02440^a^

a P<0.01 compared to the corresponding value in the control group. DM, diabetes mellitus.

RETRACTED

**Table III.** Optical density of collagen II in the disc of each group.

Group	4 weeks	8 weeks	12 weeks
Control	0.6473±0.02904	0.6039±0.03206	0.5774±0.01169
DM	0.4951±0.01540	0.3609±0.04598	0.2594±0.02365

DM, diabetes mellitus.

**Table IV.** MVD of the disc in each group.

Group	4 weeks	8 weeks	12 weeks
Control	20.80±1.048	18.96±0.910	17.28±0.716
DM	18.36±0.684^a^	15.24±1.479^a^	10.72±0.460^a^

a P<0.01 compared to the corresponding value in the control group. MVD, microvessel density; DM, diabetes mellitus.

**Table V.** AI of the notochordal cells in the disc of each group.

Group	4 weeks	8 weeks	12 weeks
Control	4.42±0.653	6.06±1.064	8.86±0.559
DM	15.92±1.403^a^	17.72±0.890^a^	23.38±1.798^a^

a P<0.01 compared to the corresponding value in the control. AI, apoptotic index; DM, diabetes mellitus.

## References

[1] Dagher Z, Park YS, Asnaghi V, Hoehn T, Gerhardinger C, Lorenzi M (2004). Studies of rat and human retinas predict a role for the polyol pathway in human diabetic retinopathy. Diabetes.

[2] Gu D, Reynolds K, Duan X (2003). Prevalence of diabetes and impaired fasting glucose in the Chinese adult population: international collaborative study of cardiovascular disease in Asia (InterASIA). Diabetologia.

[3] Hage FG, Dean P, Bhatia V, Iqbal F, Heo J, Iskandrian AE (2011). The prognostic value of the heart rate response to adenosine in relation to diabetes mellitus and chronic kidney disease. Am Heart J.

[4] Nicholas SB (2003). Advances in pathogenetic mechanisms of diabetic nephropathy. Cell Mol Biol (Noisy-le-grand).

[5] von Haehling S, Lainscak M, Doehner W (2010). Diabetes mellitus, cachexia and obesity in heart failure: rationale and design of the studies investigating co-morbidities aggravating heart failure (SICA-HF). J Cachexia Sarcopenia Muscle.

[6] Aufdermaur M, Fehr K, Lesker P, Silberberg R (1980). Quantitative histochemical changes in intervertebral discs in diabetes. Exp Cell Biol.

[7] Saito M, Marumo K (2010). Collagen cross-links as a determinant of bone quality: a possible explanation for bone fragility in aging, osteoporosis, and diabetes mellitus. Osteoporos Int.

[8] Silberberg R, Adler JH, Meier-Ruge W (1986). Effects of hyperinsulinism and of diabetes on proteoglycans of the intervertebral disc in weanling sand rats. Exp Cell Biol.

[9] Sun HL, Li CD, Wang SJ (2011). Retrospective analysis of effect of type 2 diabetes mellitus on lumbar intervertebra disc herniation. Beijing Da Xue Xue Bao.

[10] Urban JP, Smith S, Fairbank JC (2004). Nutrition of the intervertebral disc. Spine (Phila Pa 1976).

[11] Won HY, Park JB, Park EY, Riew KD (2009). Effect of hyper-glycemia on apoptosis of notochordal cells and intervertebral disc degeneration in diabetic rats. J Neurosurg Spine.

RETRACTED

[12] Feng G, Zhao X, Liu H (2011). Transplantation of mesenchymal stem cells and nucleus pulposus cells in a degenerative disc model in rabbits: a comparison of 2 cell types as potential candidates for disc regeneration. J Neurosurg Spine.

[13] Haschtmann D, Ferguson SJ, Stoyanov JV (2008). Apoptosis and gene expression of collagenases but not gelatinases in rabbit disc fragment cultures. J Neurosurg Spine.

[14] Sheikh H, Zakharian K, De La Torre RP (2009). In vivo intervertebral disc regeneration using stem cell-derived chondroprogenitors. J Neurosurg Spine.

[15] Hee HT, Chuah YJ, Tan BH, Setiobudi T, Wong HK (2011). Vascularization and morphological changes of the endplate after axial compression and distraction of the intervertebral disc. Spine (Phila Pa 1976).

[16] Wang J, Tang T, Yang H (2007). The expression of Fas ligand on normal and stabbed-disc cells in a rabbit model of intervertebral disc degeneration: a possible pathogenesis. J Neurosurg Spine.

[17] Yoon SH, Miyazaki M, Hong SW (2008). A porcine model of intervertebral disc degeneration induced by annular injury characterized with magnetic resonance imaging and histopatho-logical findings. Laboratory investigation. J Neurosurg Spine.

[18] Zhang H, La Marca F, Hollister SJ, Goldstein SA, Lin CY (2009). Developing consistently reproducible intervertebral disc degeneration at rat caudal spine by using needle puncture. J Neurosurg Spine.

[19] Weidner N (1995). Intratumor microvessel density as a prognostic factor in cancer. Am J Pathol.

[20] Ogata K, Whiteside LA (1981). 1980 Volvo award winner in basic science. Nutritional pathways of the intervertebral disc An experimental study using hydrogen washout technique. Spine (Phila Pa 1976).

[21] Rajasekaran S, Venkatadass K, Naresh Babu J, Ganesh K, Shetty AP (2008). Pharmacological enhancement of disc diffusion and differentiation of healthy, ageing and degenerated discs: results from in-vivo serial post-contrast MRI studies in 365 human lumbar discs. Eur Spine J.

[22] Edwards WT, Zheng Y, Ferrara LA, Yuan HA (2001). Structural features and thickness of the vertebral cortex in the thoracolumbar spine. Spine (Phila Pa 1976).

[23] Roberts S, Menage J, Urban JP (1989). Biochemical and structural properties of the cartilage end-plate and its relation to the inter-vertebral disc. Spine (Phila Pa 1976).

[24] Dong F, Dai K, Hou X (1995). An experimental study on the relationship between disc nutrition and disc degeneration. Zhonghua Wai Ke Za Zhi.

[25] Oki S, Matsuda Y, Shibata T, Okumura H, Desaki J (1996). Morphologic differences of the vascular buds in the vertebral endplate: scanning electron microscopic study. Spine (Phila Pa 1976).

RETRACTED

[26] Nerlich AG, Schaaf R, Walchli B, Boos N (2007). Temporo-spatial distribution of blood vessels in human lumbar intervertebral discs. Eur Spine J.

[27] Caterini R, Mancini F, Bisicchia S, Maglione P, Farsetti P (2011). The correlation between exaggerated fluid in lumbar facet joints and degenerative spondylolisthesis: prospective study of 52 patients. J Orthop Traumatol.

[28] Cho H, Park SH, Lee S, Kang M, Hasty KA, Kim SJ (2011). Snapshot of degenerative aging of porcine intervertebral disc: a model to unravel the molecular mechanisms. Exp Mol Med.

[29] Roberts S, Evans H, Trivedi J, Menage J (2006). Histology and pathology of the human intervertebral disc. J Bone Joint Surg Am.

[30] Adams MA, Freeman BJ, Morrison HP, Nelson IW, Dolan P (2000). Mechanical initiation of intervertebral disc degeneration. Spine (Phila Pa 1976).

[31] Zhao CQ, Wang LM, Jiang LS, Dai LY (2007). The cell biology of intervertebral disc aging and degeneration. Ageing Res Rev.

[32] Cheung KM, Samartzis D, Karppinen J (2010). Intervertebral disc degeneration: new insights based on ‘skipped’ level disc pathology. Arthritis Rheum.

[33] Tsutsumi S, Yasumoto Y, Ito M (2011). Idiopathic intervertebral disk calcification in childhood: a case report and review of literature. Childs Nerv Syst.

[34] Benneker LM, Heini PF, Alini M, Anderson SE, Ito K (2005). 2004 Young Investigator Award Winner: vertebral endplate marrow contact channel occlusions and intervertebral disc degeneration. Spine (Phila Pa 1976).

[35] Omlor GW, Bertram H, Kleinschmidt K (2010). Methods to monitor distribution and metabolic activity of mesenchymal stem cells following in vivo injection into nucleotomized porcine intervertebral discs. Eur Spine J.

